This article has been retracted.

# Prevalence, Mechanisms, Treatment, and Complications of Hypertension Postliving Kidney Donation

**DOI:** 10.1155/2021/5460672

**Published:** 2021-02-04

**Authors:** Stuart Deoraj, Dimitrios Anestis Moutzouris, Maria Irene Bellini

**Affiliations:** ^1^Guy's and St. Thomas' NHS Foundation Trust, UK; ^2^Azienda Ospedaliera San Camillo Forlanini, Rome, Italy

## Abstract

Living kidney donors represent a unique population of patients. Potential donors are selected based on the belief that their preoperative fitness is likely to mitigate the risks of long- and short-term harm following uninephrectomy. Studies performed on postdonation outcomes have largely focused on mortality and the risk of end-stage renal failure, but have also investigated secondary outcomes such as cardiovascular morbidity and hypertension. It has been postulated that hypertension is a possible outcome of living kidney donation. A variety of studies have been conducted to investigate the prevalence, epidemiology, mechanisms, treatment strategies, and long-term ramifications of hypertension postdonation. These studies are heterogeneous in their population, design, methodology, and outcome measures and have presented contradicting outcomes. Additionally, the absence of a well-matched control group has made it challenging to interpret and generalise the reported findings. As such, it is not possible to definitively conclude that hypertension occurs at a higher rate among donors than the general population. This article will review the evidence of postdonation hypertension prevalence, mechanisms, treatment, and complications.

## 1. Introduction

Kidney transplantation, for the majority of patients with end-stage renal failure, remains the treatment of choice of renal replacement therapy (RRT) [1] [2]. Despite the dawn of complex, patient- and evidence-directed immunosuppressive treatment, compared with deceased kidney donation, living kidney donation is significantly associated with sustainably improved long-term physical, biochemical, and psychological outcomes of the recipients [3, 4]. Regardless however, deceased donation currently accounts for over 60 percent of kidney transplantation occurring in both the United Kingdom and United States, alluding somewhat to the complexities and challenges associated with appropriate donor selection [5, 6].

A vast wealth of evidence exists on the long-term health complications associated with end-stage renal failure and dialysis, particularly regarding the effects on patient-related qualitative outcomes and cardiovascular mortality which adjusts following kidney transplantation [7–10]. The volume of high-quality literature on long-term outcomes following an elective nephrectomy from an otherwise healthy donor is comparatively scanty. This review is aimed at assessing previous literature for evidence of the long-term sequelae in living kidney donation, focusing on the onset, epidemiology, prevalence, outcomes, and burden of hypertension following donor nephrectomy.

## 2. Challenges in the Literature Review of Living Kidney Donors

Living kidney transplant donors represent a unique subset of the general population both pre- and postdonation. The process of performing a surgical procedure with the intent of harvesting a fully functioning organ from a healthy individual has historically been debated as a potentially ethical grey area, which is counterbalanced by the belief that the harm induced to the donor is negligible and comparatively outweighed by the potential benefit provided to the recipient [11].

In an ideal setting, a robust selection process for kidney donors, including preoperative counselling and physical assessment, is aimed at identifying potential donors at the peak of health and exist at the upper end of the population normal distribution curve for their age- and sex-matched peers. Following donation, they represent a cohort of healthy individuals with solitary kidneys. These characteristics make this cohort of patients inherently challenging to effectively match to control groups from the general population, even when adjusted for age and gender. Conclusions drawn from this data on the quantitative and qualitative outcomes are therefore challenging to interpret or generalise [12].

Additionally, the majority of donors are discharged from follow-up relatively quickly given the low incidence of perioperative morbidity and mortality [13, 14]. In the UK, long-term follow-up data is largely missing in these patients because their follow-up does not form part of standard clinical practice for the majority of donors.

Another major pitfall in the existing literature on donors is a lack of transparency and uniform standardisation in the selection and fitness testing of potential donors. Uncertainty regarding the parameters of fitness among donors in previous literature dramatically increases the challenges faced in generalising the findings previously reported, particularly when counselling these patients in clinic. The diagnosis of hypertension is likely to be one of the indications for longer-term follow-up of donors, a phenomenon which may introduce bias by apparently inflating the proportion of hypertensive donors who are included in studies.

It is noteworthy that biochemical evidence suggests that following nephrectomy, the circadian rhythm of the renin-angiotensin-aldosterone system (RAAS) undergoes significant remodelling [15]. Inconsistencies in the measurement methodology and time may well skew the findings of these longitudinal studies. A further issue identified includes the heterogeneity in ethnicity among study groups, which significantly impacts generalisability to clinical practice in multiethnic societies [16, 17].

In addition to the above, despite the apparent health of potential donors, the demographics of these patients is a key aspect which must be considered. The vast majority of studies on the topic of hypertension as a long-term outcome of living kidney donation do not discriminate between related and unrelated donors. Epidemiological data suggests that renal disease is predominantly seen in patients with diabetes and cardiovascular disease. These primary illnesses are also prevalent among lower socioeconomic groups. Living-related or partnered donors may share similar genetic and socioeconomic traits as their recipients and, as such, may be exposed to similar cardiovascular risks [18–20].

What is also unclear from the literature is the blood pressure outcome of the recipients specifically from donors who develop de novo hypertension. Given that the blood pressure profile in transplant patients is heavily dependent on the phenotype of the transplanted kidney, hypertension among recipients may allude to an underlying process specific to the donor, rather than simply uninephrectomy.

Understandably, controlled studies have yet to accomplish matching which accommodates beyond age and sex and also considers the role of shared socioeconomic and genetic factors in prognosis among this unique cohort. Alongside this, the qualitative aspect of the psychological stressors associated with living kidney donation has only recently become apparent and represents yet another aspect of hypertension prediction which has not been explored or appropriately matched in previous trials and studies [21–24].

## 3. Prevalence of Postdonation Hypertension in Living Kidney Donors

The literature regarding the incidence and prevalence of hypertension in the years following living kidney donation is characterised predominantly by inconsistency in study design and outcomes [12]. While the majority of these papers assessed kidney donors retrospectively as a cohort, little data is presented on predonation clinical parameters including smoking status, cardiovascular fitness, or family history.

Among these studies, there is wide variability in the time point postdonation at which blood pressure is assessed and reported. Exclusion criteria vary between studies, occasionally, including individuals with predonation hypertension or subgroups with statistically significant variability in their predonation blood pressure [16, 25]. The lack of cohesiveness in the donor cohorts of reported literature drives a significant degree of uncertainty in the generalisability of the data. Often the cohort size within these studies is small, hampered by loss to follow-up, in itself a form of bias as highlighted above [26, 27]. In these studies, there is significant variation of donor characteristics. Particularly relevant to the smaller studies, comparison against age- and sex-matched controls becomes challenging for subgroup analyses.

The definition and robustness of a diagnosis of hypertension vary, with some studies relying heavily on medication lists and only one study investigating the use of ambulatory blood pressure measurements (ABPM) in the diagnosis of hypertension. Holscher et al. assessed over 41000 patients with a relatively short follow-up period of two years divided into blocks from which statistical estimation was used to arrive at a diagnosis of hypertension given significant data gaps [19]. They identified an exponential rise in hypertension prevalence at two years, but based their diagnosis on centre-reported data rather than objective measures of blood pressure. Comparatively, Yadav et al. conducted a prospective observational study on a smaller group of only 51 patients of whom most were women who were followed up for only three months, but utilized ABPM [18, 27]. Another study by Holscher et al., drawn from the American WHOLE-Donor trial, relied heavily on the use of self-reported diagnosis of hypertension and did not use baseline objective measures of blood pressure in the calculation of postdonation prevalence.

This study reported a hazard ratio of 1.19 (*p* = 0.04), for the outcome of self-reported hypertension among donors compared to healthy controls [28]. Preexisting trial data from a population study was used as a surrogate marker for the outcome of hypertension among the general population. It was weighted for age, race, and sex, but was not validated to match more detailed health characteristics of the donor population. Among the studies, the average age at donation varies significantly, allowing wide margins of error [25, 29]. Additionally, as discussed previously, the absence of a truly comparable control group which meets an adequate threshold from which to draw conclusions about the natural history of living kidney donation creates significant obscurity in the understanding of the study findings.

The single largest landmark controlled study assessing long-term outcomes in 1900 donors compared to a group of 30000 age-, gender-, BMI- (body mass index-), and blood pressure-matched controls, by Mjøen et al., informs the counselling of long-term renal failure outcomes in potential kidney donors [26]. This study did not report on hypertension prevalence, but assessed all-cause and cardiovascular mortality. The adjusted hazard ratio for all-cause mortality following kidney donation, once adjusted by multiple imputation, was 1.4 (p = 0.03). Of note, this value is widely different from the unadjusted hazard ratio of 3.18 (p < 0.001), suggestive of the misleading potential of inappropriate control matching. Other types of studies including projected analyses using simulation software suggest a significantly higher prevalence of hypertension should be expected among donors compared to controls, but the reliability of these types of studies remains undermined by the problematic nature and uncertainty of predicting late events [30].

It is unsurprising, given the above, that studies assessing the prevalence of hypertension following elective uninephrectomy in healthy donors have highly variable reported outcomes compared to either controls or age- and sex-matched individuals from general population epidemiological studies. Studies which have proposed that there is a significant risk of developing increased blood pressure following donation are faulted by poor design, the absence of a meaningful control group, and small sample size [2, 12, 16, 25, 31, 32].

Among these studies, Thiel et al. reported on a prospective Swiss cohort of 1214 donors with a follow-up of 10 years and identified that compared to the Framingham data of age- and sex-matched controls, the risk of hypertension at 1 year was triplicated by kidney donation compared to the general population [25]. This study reported that the predicted risk of developing hypertension compared to healthy controls was 3.64 (*p* < 0.001). Despite the prospective design of this study, significant data gaps requiring sensitivity analyses were employed. 26% of patients were lost to follow-up, and this study design did not exclude patients from analysis who had significantly higher predonation systolic blood pressure.

Comparatively, similar limitations can be identified among studies suggesting that the prevalence of hypertension is equivalent to or less than that expected of the general population [17, 33–40]. Sanchez et al. performed a robust analysis of 3700 donors matched to controls based on NHANES epidemiological studies and reported on the prevalence of hypertension among predominantly Caucasian donors, relying heavily on donor self-reporting. The matching performed in this study did not include robust exclusion criteria among the NHANES cohort. As such, the data reported on population statistics among age-matched groups, but lacked an intensive subgroup consisting of controls with other baseline features that would make them more comparable to donors. They identified that the prevalence of hypertension was significantly less than that expected of age-matched controls, a finding which is challenging to generalise given the limitations above. This study performed subgroup analyses which identified that the incidence of hypertension is highly dependent on the accumulation of risk factors in addition to uninephrectomy. Of note, the patients who developed postdonation hypertension were categorically distinct from those who did not. They were older, tended to be smokers with higher BMIs and higher creatinine and cholesterol measurements postdonation. The mean starting blood pressure in patients who developed hypertension was higher than that of those who did not develop hypertension after 50 years. Additionally, the slope of blood pressure incrementation over time was steeper for those who developed hypertension by a small but statistically significant margin of 0.9 mmHg/decade (*p* < 0.0001).

Over a period of forty-five years, a progressive rise in blood pressure was identified among all patients. In those who achieved hypertension, a rate of increase of 2.9 mmHg per decade in systolic pressure was recorded, compared to a rate of increase of 2 mmHg per decade among nonhypertensive patients. A progressive rise in blood pressure has previously been demonstrated among adults and has been attributed to age-related phenomena, genetic and environmental factors, and vascular remodelling.

The underlying characteristics of these patients were distinct, with higher end blood pressure identified among persons with higher BMI (*p* < 0.001), smokers (*p* < 0.001), older donors (*p* < 0.001), lower estimated glomerular filtration rate (eGFR) (*p* < 0.001), and first-degree relatives of the recipient (*p* < 0.001). Additionally, this study identified that the risk of hypertension was exacerbated by the cumulative presence of these synergistic risk factors.

Among the most robust studies, Saran et al. suggested that a group of donors matched against epidemiological data from the NHANES III and Whickham studies showed a statistically significant trend towards a higher prevalence of hypertension over time, particularly past the age of 60 [32]. Given that this publication related to a small cohort of patients assessed between the years 1963 and 1982, the findings reported in this paper are challenging to apply to current clinical practice [32].

A key meta-analysis of published studies of donors by Boudville concluded that over time, an average rise of 5 mmHg in systolic blood pressure was observed in donors as opposed to controls. Having assessed forty-eight papers accumulating greater than 5000 patients, the authors mentioned that certainty of this finding was consistently hampered by poor study design, incomplete follow-up, and small individual studies with variable end points and exclusion criteria [12].

One consistent finding throughout the literature is the certainty that the presentation of hypertension is not a unanimous phenomenon. Recurrently, a tendency towards hypertension was observed to predominate in ethnic minorities, donors with higher BMI, men, and older donors longitudinally over time [2, 19, 34, 35, 41]. While this effect is likely on par with the expected blood pressure rise within this group over time, an inflated prevalence among donors is possible, but challenging to quantify or prove conclusively given the current body of evidence. An important consideration however includes a small study by Doshi et al., conducted in 100 African-American donors in which all donors were genotyped for APOL1 gene mutations and stratified by risk [42]. Although homozygous donors are believed to be the most pathogenic genotype of APOL1, the study identified that the risk of postdonation hypertension among these patients was equivalent to lower risk genotypic variations.

The few studies which were adequately powered to assess subgroups within the donor cohort also concurred that hypertension was more prevalent among relatives and partners of kidney transplant recipients, indicating a social or genetic phenomenon which may contribute to the outcomes identified [19].

It is noteworthy that other human studies that may provide insight into the prevalence of hypertension include the subgroup analyses of patients with renal tumours under the age of 75 who have either radical nephrectomy or nephron sparing therapy. As directly comparable groups, there is a propensity towards hypertension among persons with radical nephrectomy [43].

In contrast to the nature of human studies, a clinico-biochemical controlled study published in an animal model of uninephrectomy with follow-up over a period of 18 months supported the finding of a statistically significant prevalence of hypertension among male nephrectomised rats vs. nonnephrectomised males. In this study, renal salt handling and diuresis appeared significantly better among female rats compared to male rats. Despite the pitfalls of animal studies, the findings of this paper serve as a modelling tool in the absence of a clear answer among human studies [44].

Overall, it is reasonable to conclude from the literature that the prevalence of hypertension among donors occurs likely, at least at the same rate as expected among matched controls for the first decade following donation. Beyond this time frame, the data is increasingly unclear because of significant gaps in follow-up. This rate is also unlikely to be uniform among all donors, but may be dependent on coincidental modifiable and nonmodifiable risk factors including race, age, gender, predonation blood pressure, and BMI.

## 4. Potential Mechanisms of Postdonation Hypertension in Living Kidney Donors

Hypertension is frequently associated with chronic kidney disease via complex, multistep mechanisms which include water and salt handling, endothelial dysfunction, RAAS activation, and nervous system hyperactivity [46]. To a degree, derangement of these steps is likely primed by preexisting illnesses, which are largely absent among healthy living kidney donors compared to the general population.

A popular explanation for hypertension among living kidney donors refers to the “nephron number” theory. This theory explains that the risk of developing hypertension is inversely proportional to the active number of nephrons (Figure 1) [47]. The mechanism by which nephron number contributes to hypertension is poorly understood. While this phenomenon has been identified in rat models, the true incidence and mechanism of hypertension among living kidney donors remain unclear and are likely cushioned by an adaptive response in the remaining kidney. A summary of the current evidence is provided in Table 1.

Following kidney donation, structural analysis of the remaining kidney suggests a number of important adaptive changes. This includes firstly a significant hypertrophy and endowment of nephron-rich parenchyma. Second, adaptive benign hyperfiltration and an increased cardiac output have been observed [48–50]. These mechanisms suggest that nephron number may not be a significant determinant of hypertension among donors.

This raises the possibility of a “second hit” phenomenon, which relies on a superadded insult following nephrectomy [48]. What is clear from the literature is that living kidney donors are heterogeneous in their baseline characteristics. Of note, a higher baseline blood pressure, elevated BMI, older age, and certain ethnic origins augment the trajectory of blood pressure postdonation. This suggests that among healthy individuals who have undergone an elective uninephrectomy, the generation of hypertension is driven by specific mechanisms which interact with the adaptive cardiovascular remodelling, rather than directly related to donation.

Animal models have provided evidence of reduced effectiveness of salt handling and have demonstrated blood pressure in uninephrectomised animal models to be salt sensitive [51]. In this study of 3-week-old rats which were randomised to either sham or uninephrectomy operations, a period of 6-8 weeks of study was employed with a second layer of randomisation to either high or normal salt diets. This study demonstrated that the incidence of hypertension was the greatest among predominantly male, uninephrectomised rats which were exposed to high salt intake. Additionally, a relative 11 beta-hydroxylase deficiency identified in rat models potentially represents an alternate explanatory mechanism [52]. In this study, 8-week-old rats were randomised to either sham or uninephrectomy operations followed by a period of monitoring aldosterone, protein, and corticosteroid metabolites. These models suggest that the generation of hypertension is a separate event from simply structural glomerular damage and indicates that uninephrectomy is not directly causal of hypertension, but instead results in downstream mechanisms which augment blood pressure [53].

Given the evidence of heterogeneity in the onset of hypertension among donors and an apparent prevalence of hypertension, particularly among men, Hispanic and Black donors, the onset of hypertension following kidney donation is likely only in part related to the structural and functional adaptations. There is likely a genetic or epigenetic component which fulfills the “second hit,” which is yet to be fully elucidated.

## 5. Complications of Postdonation Hypertension in Living Kidney Donors

In the general population, uncontrolled hypertension has a strong causal effect on the outcomes of end organ damage, particularly including cardiovascular mortality, the burden of polypharmacy, end-stage renal failure, and proteinuria [54]. Similar to above, the natural history of hypertension in living kidney donors is not fully elucidated, and the outcomes reported in the literature are marked by inconsistency. Some studies suggest that long-term outcomes of uninephrectomy are beneficial to mortality and that there is no difference from the general population, while others suggest a significant trend towards increased morbidity and mortality.

Mjøen et al. reported that the cumulative all-cause mortality and chronic kidney disease are inflated among donors [45]. The role of hypertension itself as a factor in this propensity is however unclear. This study matched over 1500 donors against 30000 healthy controls according to a variety of criteria. The study matching protocol was highly robust and included careful exclusion of controls based on health characteristics that would have prevented them from becoming living kidney donors. Of note, the control group had strict BMI, blood pressure, and age exclusion criteria. Consequently, the control group employed was likely highly comparable to the donor population. The study reported that the hazard ratio of adjusted all-cause mortality among donors was 1.4 (*p* = 0.03). Additionally, the adjusted Cox regression analysis end-stage renal disease after multiple imputation was 11.38 (*p* ≤ 0.001) for donors compared to controls. Importantly, this subgroup analysis compared 31 patients to 34522 controls. Despite its strong statistical significance, the validity of this finding is challenging to translate into practice.

Epidemiological data suggests cardiovascular disease to be a global pandemic directly associated with mortality [45]. In contrast to this, long-term studies have suggested malignancy to outrank cardiovascular disease as a leading cause of death in living kidney donors [55]. A number of studies have gone on to postulate that the role of hypertension is likely an aspect of adaptive physiological change, but accept that there is adequate uncertainty about long-term outcomes which is fostered by the study limitations [56–60].

It is well recognised from robust cardiovascular studies that following uninephrectomy, significant physical adaptations occur, inclusive of cardiac remodelling characterised by a statistically significant increase in ventricular mass among donors compared to controls [58]. The role of this however may prove to be representative of adaptive phenomena rather than immediately pathogenic.

The evidence suggests that cardiovascular mortality in donors is no different from the general population in the first decade postdonation, suggesting that cardiac remodelling and cardiovascular adaptations may not carry the weight of clinical significance [61]. Additionally, multiple logistic regression has identified that the onset of hypertension correlates poorly with glomerular filtration rate, smoking, and proteinuria [33].

It is noteworthy however that these finding may be cushioned by the cherry-picking bias imposed on the literature by having pristinely healthy donors compared to the age- and sex-matched population, making generalisation of these findings largely misleading.

## 6. Treatment and Prevention of Postdonation Hypertension in Living Kidney Donors

Living kidney donation is associated with a robust series of assessments and counselling of potential donors. Predonation assessment and counselling need to develop on par with the developing awareness of the downstream sequelae of kidney donation including the physical and psychological elements. While there are studies assessing the risk of depression following kidney transplantation, there is undoubtedly a coexistent psychosocial benefit of kidney transplantation. These psychosocial elements and their outcome on the physical well-being of donors are yet to be unpicked. A propensity towards hypertension has been identified within certain subgroups within the donor population which may or may not have subsequent knock-on effects on cardiovascular mortality. As such, appropriate kidney donation must be accompanied by robust screening of potential donors for hypertension and cardiovascular mortality. These should not necessarily be barriers to donation, but should be used to inform potential donors of risks in a holistic way.

The evidence suggests that uninephrectomy is not clearly a risk factor for the development of de novo hypertension for all donors. The outcome of hypertension appears to be the end result of the synergistic effects of kidney donation with modifiable and nonmodifiable risk factors. As such, predonation counselling should include a risk calculator in order to provide potential donors with evidence-based decisions.

The development of hypertension and cardiovascular mortality, similar to that of the general population, is likely driven by a combination of modifiable and nonmodifiable factors. Donors should be counselled about salt restriction and monitoring of blood pressure at home. Given the uncertainty presented in the data on the long-term sequelae of hypertension among donors, it is unclear what target blood pressure should be recommended.

Modifiable risk factors, such as smoking and elevated BMI, that impede the health and well-being of patients and appear to contribute to hypertension should be addressed, although these should not be considered per se a contraindication to donate [62]. Older donors should be counselled on the apparent increased likelihood of developing hypertension. Additionally, given the finding of increased cardiovascular and all-cause mortality over time, longer follow-up should be instituted for donors as part of clinical practice, particularly among men, those who are older, those who belong to ethnic minority groups, those who smoke, and those with higher BMI at the time of donation [26]. The median time to diagnosis of hypertension according to Sanchez et al. was 15 years. As such, long-term follow-up for these late cardiovascular events is required.

It is worth noting that by standard description, kidney donors do not fall into a category that is truly comparable to age- and sex-matched controls in the general population. Given that hypertension may well represent the end product of an adaptive process in an individual who is apparently at no greater risk of cardiovascular mortality, some studies have postulated that a reasonable degree of permissive hypertension is likely appropriate, rather than intensive blood pressure control [63].

Further study is required to delineate the prevalence of hypertension among kidney donors, particularly given the changes in approach to identification, selection, and management of donors. One such study which may shed light on the role of uninephrectomy on the outcome of hypertension may include an analysis of recipients from donors who develop postdonation de novo hypertension. This may indicate a donor-specific phenomenon responsible for the genesis of hypertension.

## 7. Conclusion

There remains significant uncertainty regarding the prevalence, pathophysiology, complications, and management of hypertension following living kidney donation. It is unclear whether or not there is a significant risk of hypertension in donors compared to the general population. It appears clear from the evidence that the propensity for hypertension is a heterogeneous phenomenon which affects donors to different degrees and may be related to ethnicity, age, time from transplant, and BMI.

This data suggests that hypertension occurs following kidney donation most readily among certain subgroups of patients, particularly those with higher BMIs, smokers, and those with higher predonation creatinine and blood pressures. In the future, this could inform decision-making when assessing potential living donors, but requires further work.

The mechanisms driving hypertension are likely to be inexorably linked with renal salt handling and a deficiency in nephron number contextualised to individual characteristics and are similarly likely to be part of an adaptive process following uninephrectomy. The long-term sequelae of hypertension among donors remain unclear.

Overall, there may be a small to modest increase in blood pressure postdonation, which is more apparent in certain subgroups of donors, but the validity of these findings has consistently been hampered by the absence of a meaningful control group, significant bias, small sample size, retrospective design, and poor follow-up. Additionally, this propensity to developing de novo hypertension is likely reliant on a complex interplay of nephrectomy contextualised to individual risk factors. Among these patients, the risk of developing hypertension appears to result in significant cardiovascular remodelling. These outcomes do not appear at present to have a significant bearing on clinical outcomes, but further long-term data is required to resolve this matter conclusively.

## Figures and Tables

**Figure 1:** Demonstrating potential mechanisms of de novo hypertension in kidney donors.

**Table 1:** Highlighting the findings of key studies and their respective strengths and limitations.

Authors	Sample size	Study design	Length of follow-up	Comparator	Measure	Key findings	Strengths	Limitations
Hakim et al. [16]	*N* = 52	Prospective study design	10 years	Age- and sex-matched controls from general population	Incidence of diastolic hypertension over time	60% vs. 17%		Age- and sex-matched control from the general population and from inpatient population Small sample size
Yasumura et al. [17]	*N* = 247	Prospective observational study design	18 months–16 years	Matching not performed	Hypertension recorded as an outcome	2.4%	Moderate sample size Long posttransplant follow-up	No matched control groups Only Japanese patients were included
Abomelha et al. [18]	*N* = 200	Prospective observational study	3, 6, and 12 months postdonation	Matching not performed	Hypertension recorded from notes	2.9%	Moderate sample size	No matched control groups Short follow-up period
Holscher et al. [19]	*N* = 41260 patients	National cohort study	Up to 2 years postdonation	Matching not performed	Hypertension recorded from notes	3% of donors at 2 years; higher risk identified among men, older donors, and those with higher BMI	Large sample size Heterogeneous group of donors	No matched control groups Relatively short follow-up Hypertension not clearly defined Incidence estimates used for missing data
Sanchez	*N* = 4296	Observational, longitudinal cohort study	6, 12, and 24 months and then every 3 years between 1963 and 2014	Matching performed against population study NHANES				Predominantly Caucasian donors
Thiel et al. [25]	*N* = 1214 Swiss transplant cohort	Prospective observational study	10-year follow-up	Patients were not individually matched. A hypertension risk score was generated and compared to an expected value derived from the Framingham hypertension risk.	Hypertension defined as SBP > 140 and DBP > 90	Predicted risk of developing hypertension increasing by 3.64 (*p* < 0.001) using the Framingham calculator	Large sample size Hypertension clearly defined	The rate of smoking and family history of hypertension were assumed variable. Normotensive patients with high end of normal predonation blood pressure were not excluded or adjusted for.
Bhowmik et al. [29]	*N* = 51	Prospective observational study	3-month follow-up	Matching not performed	Hypertension clearly defined using ambulatory blood pressure measurements	No statistically significant increase in ABPM pre- vs. postnephrectomy	The use of ABPM to demonstrate blood pressure changes	Small sample size Short follow-up Lack of matching to an appropriate control
Holscher et al. [28]	*N* = 1295 Weighted control group *n* = 8233	Observational case-control study	6-year follow-up	Matching was made against healthy nondonors drawn from large coexisting trials and weighted for age, race, and sex.	Hypertension was defined as a self-reported outcome.	Hazard ratio of developing hypertension = 1.19 (*p* = 0.04)	Large cohort study Matching performed against young, healthy nondonors	Relied on self-reporting Weakly significant statistical findings
Saran et al. [32]	*N* = 75 (47 after exclusion)	Observational study	10-year follow-up	The prevalence of hypertension was compared to data drawn from the Whickham and NHANES III population studies.	Hypertension was defined as SBP > 140 and DBP > 90.	In the over 55 age group, the prevalence of hypertension was greater than the expected value from NHANES III and Whickham	Hypertension clearly defined Long study follow-up	Population studies used rather than matching Small sample size Predonation hypertensives were not excluded.
Gossmann et al. [33]	*N* = 152 Control *N* = 7101	Case-control observational study	Assessed individual cases at a time point postdonation up to 28 years	Compared cases to data drawn from a large German cohort study Matched to age and gender	Blood pressure was compared as a variable rather than a hypertensive diagnosis.	Prevalence of hypertension significantly lower among donors than nondonors (*p* < 0.01)	Case-control design Large study Multiple time points postdonation for longitudinal information	
Mjøen et al. [45]	*N* = 1901 Controls *n* = 32621	Case-control study	Assessed cardiovascular death and risk of end-stage renal disease in kidney donors vs. control	Population data from the HUNT1 survey of Norway was used. Patients excluded based on health and age criteria. Robust matching to donor cohort	Risk of death from cardiovascular or all-cause assessment Hazard ratio = 1.01 (*p* = 0.03)		Large study Well matched to the control group Follow-up as long as 26 years postdonation	

## Abbreviations

ABPM: Ambulatory blood pressure measurements
BMI: Body mass index
eGFR: Estimated glomerular filtration rate
RAAS: Renin-angiotensin-aldosterone system
RRT: Renal replacement therapy.
